# Nursing Countermeasures of Continuous Renal Replacement Treatment in End-Stage Renal Disease with Refractory Hypotension in the Context of Smart Health

**DOI:** 10.1155/2022/2382458

**Published:** 2022-08-10

**Authors:** Liya Ma, Jianli Guo, Hongwei Sun, Nan Li, MeiXuan Lv, Bing Shang

**Affiliations:** Endoscopy Center, The First Affiliated Hospital of Qiqihar Medical University, Qiqihar, 161006 Heilongjiang, China

## Abstract

This work is aimed at exploring the nursing strategies and effects of continuous renal replacement therapy (CRRT) for end-stage renal disease (ESRD) with refractory hypotension under the background of smart health. 40 ESRD patients with refractory hypotension who received CRRT treatment were enrolled as the research objects and were randomly rolled into the intervention group and the control group, with 20 cases in each group. Patients in the control group received routine nursing, and those in the intervention group received individualized nursing. The incidence of hypotension, dry body weight, serous cavity effusion, renal function indicators (blood urea nitrogen (BUN) and creatinine (Cre)), and patient satisfaction were compared between the two groups. The results showed that the probability of hypotension in the intervention group was 9.38%, which was lower than that in the control group (34.38%). The probability of early termination of dialysis in the intervention group was 0%, which was lower than that in the control group (18.75%), and the difference was statistically significant (*P* < 0.05). The decreases of BUN and Cre in the intervention group were significantly greater than those in the control group, and the differences were statistically significant (*P* < 0.05). The proportion of water growth less than 10% during dialysis in the intervention group was 98.44%, which was greater than that in the control group (93.45%), and the difference was statistically significant (*P* < 0.05). The ultrafiltration volume after dialysis in the intervention group was 2850 ± 400 mL, which was greater than that in the control group 2350 ± 350 mL. After intervention, the proportion of patients with pleural effusion in the intervention group was 10% less than that in the control group (20%), and the difference was statistically significant (*P* < 0.05). The satisfaction rate of the intervention group was 97.66%, which was higher than that of the control group (65.63%). In conclusion, individualized nursing was more helpful to the recovery of ESRD patients with refractory hypotension treated with CRRT than routine nursing.

## 1. Introduction

End-stage renal disease (ESRD) refers to a disease in which chronic kidney disease develops to the end stage, with changes in renal structure and substantial loss of renal function, also known as uremia [1]. Chronic kidney disease is divided into 5 stages. When the glomerular filtration rate of patients in stage 5 is maintained at a level of less than 15 mL/(min.1.73 m^2^), it can be diagnosed as ESRD. According to relevant statistics, the probability of chronic kidney disease in China can reach 10.8%, that is, the number of chronic kidney disease patients is about 130 million, of which about 3 million will develop ESRD [2]. ESRD is extremely detrimental to the patient's body and mind. The current treatment for ESRD patients is mainly renal replacement therapy, namely, hemodialysis, also known as blood purification [3]. Hemodialysis is a treatment method in which the patient's blood is drained to the outside of the body, the toxins in the blood are removed through a filtering device, and then, the blood is returned to the patient's body. In this process, the blood has to undergo extracorporeal circulation. Therefore, it is very important to disinfect and sterilize the relevant instruments and ensure the sterility of the operating environment to prevent blood infection. At the same time, the extracorporeal circulation of blood is established on the basis of our artificial construction of access, so the establishment of vascular access before hemodialysis is the first important preparation work. During the dialysis, medical staff should also pay attention to ensuring the smoothness of the access, to prevent the pipeline from being damaged due to human factors, or to block the access by coagulation, which will affect the dialysis effect [4]. Hemodialysis, as a widely used clinical treatment method with outstanding therapeutic effect, prolongs the life of countless kidney disease patients. However, long-term hemodialysis will also be accompanied by certain side effects. Common side effects experienced by patients includes the following aspects. Firstly, the patients may suffer from dialysis imbalance syndrome. This is because there is a significant gradient difference between the plasma osmotic pressure and the osmotic pressure of the brain, resulting in intracranial edema and high pressure causing nausea, vomiting, dizziness, and headache. Secondly, hemodialysis patients will have allergies in the early stage. Some patients are allergic to dialyzers or dialysate and may experience rashes and fever. In severe cases, chest tightness, difficulty breathing, and palpitation may occur. Thirdly, early side effects may cause muscle cramps. Fourthly, patients may have conditions that can lead to hypotension or high blood pressure. Fifthly, there will also be infections, which are rare now, and sometimes contagious hepatitis C and hepatitis B. Sixthly, patients on long-term dialysis will have carpal tunnel syndrome, or chronic osteoarthropathy, and other manifestations of dialysis-related amyloidosis. Seventhly, hemodialysis patients may also experience anemia or malnutrition. Finally, cardiac problems may occur, such as heart failure, arrhythmia, or complications such as vascular calcification [5, 6]. Among them, the probability of hypotension caused by dialysis is about 20%-40% according to statistics. However, due to the difference of each person's constitution and the ability to adapt to hemodialysis, the probability of hypotension in some patients can reach 50%-70% [7]. In the existing research, targeted treatment measures for patients with hypotension during dialysis are as follows. Firstly, it should identify the etiology. The causes of hypotension in dialysis patients include hypovolemia, decreased peripheral blood flow resistance, heart problems, malnutrition, and dialysis-related infections. Secondly, it should cooperate with the doctor to look for the specific reasons actively and carefully, and sometimes, the reasons may interact at the same time. Thirdly, it should have a reasonable diet, ensure calories and energy, and maintain a good nutritional state. Long-term salt prohibition is not advisable. Fourthly, it should evaluate the dry body weight well and avoid excessive dialysis dehydration. Fifthly, it should protect the heart function, and pericardial effusion needs to be dealt with in time. Sixthly, drugs that raise blood pressure are effective for some patients. Seventhly, refractory hypotension, such as amyloidosis and severe failure, are difficult to respond to various treatments, so that hemodialysis cannot be performed, and peritoneal dialysis can be changed [8]. Continuous renal replacement therapy (CRRT) is mainly a blood purification treatment method. It is performed continuously for several hours or nearly 24 hours a day to relieve the pressure of kidney metabolism and purification and reduce the burden on organs [9]. The working principle of this technology is to imitate the filtration function of the glomerulus, using a semipermeable membrane filter to help remove water and solutes from the blood, and to separate the substances needed by the body from the waste substances that are metabolized. Next, it can import the substances needed by the body into the body to maintain the balance of electrolytes in the body and the normal operation of the body [10]. While performing blood filtration, it can also help eliminate inflammatory mediators in the blood, improve the patient's physical condition, reduce the chance of infection and concurrent inflammation, and improve the function of the autoimmune system. At the same time, regular blood purification can maintain the overall physical state of the patient. It is mainly suitable for severe kidney, liver, heart, and other organ diseases, such as acute renal failure, uremia, hepatic encephalopathy, acute pancreatitis, and congestive heart failure. It can reduce the burden on the organs and maintain the function of the organs. It can also be used to treat autoimmune system diseases, such as sepsis and systemic inflammatory response syndrome, to help inflammatory factors to be excreted from the body, so as to reduce the damage to organs caused by the disease [11, 12].

Until now, the nursing model of some hospitals has tended to be standardized, so that patients follow the same standard for postoperative recovery plans. Although such a nursing model can have a clear standard specification, it is difficult to guarantee the surgical effect of patients [13]. But in fact, each patient is an independent individual, and their psychological situation, living environment, eating habits, etc. are different. If these individual differences are not taken into account, and only a set of standards is used to require them, it will be difficult for some patients to meet the standard requirements, and the effect of surgery will naturally be greatly reduced. Standardized care requirements can ensure patient safety, while individualized care can lead to better surgical outcomes [14]. Individualized care is not just about designing recipes based on taste preferences, but about gaining a deep understanding of the patient's heart and living environment [15]. For example, psychological counselling is carried out according to the patient's situation, and a psychological intervention plan is formulated according to his reaction. Understand the patient's usual living habits, in addition to behaviors that have a negative impact on the effect of surgery, should try to adapt to these habits when formulating a recovery plan, so as to reduce the patient's resistance to the recovery plan. At the same time, the recovery status and quality of life of patients are regularly and objectively assessed, and the plan is adjusted in time [16]. Therefore, the routine nursing and nursing strategies (i.e., individualized nursing) were adopted for ESRD patients with refractory hypotension using CRRT in this work. By comparing and observing the hypotension occurrence, dry body weight, serous effusion, blood index, nursing satisfaction, and other performances of patients under the two nursing strategies, the effect of nursing strategies can be judged.

## 2. Materials and Methods

### 2.1. Experimental Subjects

40 ESRD patients with refractory hypotension who received CRRT in The First Affiliated Hospital of Qiqihar Medical College from 2019 to 2021 were enrolled as the research subjects, including 21 males and 19 females. The age ranged 22-75 years old, with the mean age of 57.13 ± 9.75 years old. The 40 subjects were randomly rolled into the intervention group and the control group, with 20 cases in each group. There were 12 males and 8 females in the control group, while there were 11 males and 9 females in the intervention group. The experiment had been approved by the Medical Ethics Committee of The First Affiliated Hospital of Qiqihar Medical College, and the patients and their families understood the research content and methods and signed the corresponding informed consent.

Inclusion criteria were set as follows: (I) patients who were diagnosed according to ESRD diagnostic criteria, (II) patients whose systolic blood pressure (SBP) before dialysis was less than 100 mmHg or MAP decreased by more than 20 mmHg during dialysis, and (III) patients with complete clinical data.

Exclusion criteria were defined as follows: those with cardiac dysfunction, those unable to complete the experimental process, and those with incomplete clinical data.

### 2.2. Experimental Methods

The patients in the intervention group received individualized nursing on the basis of CRRT. Individualized nursing measures were tailored according to the complications that were prone to occur in patients with ESRD with refractory hypotension during treatment. The subjects in the control group received routine nursing on the basis of CRRT. The occurrence of hypotension, weight change, and nursing satisfaction in each dialysis group were recorded during the three months of nursing intervention (a total of 640 times of dialysis in the intervention group and in the control group). In addition, the performance of ultrafiltration volume, serous effusion, and renal indicators before and after three months of intervention were also recorded. Through comparative analysis, the effect of individualized nursing strategies can be determined. The specific experimental process was shown in Figure 1.

### 2.3. Flowchart of CRRT

CRRT, also known as bedside hemofiltration, is a long-term continuous extracorporeal blood purification therapy for 24 hours or nearly 24 hours a day to replace damaged kidney function, as shown in Figure 2.

### 2.4. Nursing Measures

Nursing routine procedures included standardized disinfection treatment, operation to ensure sterile state, and regular observation and recording of clinical indicators of patients.

Compared with routine nursing, scientific countermeasures are applied for the individualized nursing according to the specific situation of the patient, not only the nursing of the condition but also the psychological nursing.  Table 1 showed the specific content of individualized nursing [17].

### 2.5. Observation Indicators

The observation indicators included the incidence of hypotension, early dialysis end rate, ultrafiltration volume, weight change, BUN, Cre, serous effusion, and nursing satisfaction.

Diagnostic criteria for hypotension during dialysis: a decrease in SBP > 20 mmHg or a decrease in MAP > 10 mmHg accompanied by hypotension symptoms such as headache, nausea, and sweating.

Target ultrafiltration volume = the body mass before dialysis − dry body mass + fluid return volume at the end of dialysis,

The ultrafiltration volume after dialysis = the actual ultrafiltration volume displayed by the dialysis machine at the end of dialysis.

In the early end of dialysis, the patient's dialysis time was less than the length of dialysis prescribed by the doctor.

### 2.6. Statistical Methods

SPSS 20.0 was used for statistical analysis, count data were expressed as frequency and percentage, and *χ*^2^ test was used for comparison between groups. Measurement data were expressed as mean ± variance, and independent samples *t* test was used for comparison between groups. *P* < 0.05 meant difference was statistically significant.

## 3. Results

### 3.1. Basic Data

There was no significant difference between the two groups in age, gender, course of disease, and the number of weekly dialysis (*P* > 0.05). The patients in two groups were comparable, as shown in Table 2.

### 3.2. Comparison on Incidence of Hypotension

The incidence of hypotension and the early termination rate of dialysis between the two groups were obviously different (*P* < 0.05). In the 640 times of dialysis, the probability of hypotension was 9.38% in the intervention group and 34.38% in the control group. The probability of hypotension in the intervention group was lower (*P* < 0.05). The probability of early termination of dialysis due to hypotension was 0% in the intervention group, which was much lower than 18.75% in the control group (*P* < 0.05). The specific results were shown in Table 3.

### 3.3. Comparison of Renal Function Indicators

The BUN and Cre levels of the two groups of patients before and after the intervention were observed, and the results were given in Tables 4 and 5. The BUN and Cre levels of the two groups of patients were decreased to a certain extent compared with those before the intervention (*P* < 0.05). The two indicators in the intervention group decreased significantly more than that in the control group.

### 3.4. Comparison of Body Weight Changes

The weight changes of the two groups before and after the intervention were compared, and the results were given in Table 6. Before intervention, the proportion of water growth less than 10% in the intervention group during dialysis was 93.75%, and the proportion in the control group was 91.72%, showing statistical difference (*P* > 0.05). After the intervention, the proportion of water growth less than 10% in the intervention group during dialysis was 98.44%, and the proportion in the control group was 93.45%, showing statistically great difference (*P* < 0.05). The number of patients with water growth less than 10% during dialysis before and after the intervention, the number of patients in the intervention group was significantly more than that in the control group.

### 3.5. Comparison of Target Dialysis Ultrafiltration Volume before Dialysis and Ultrafiltration Volume after Dialysis

The target dialysis ultrafiltration volume before dialysis was compared between the two groups, and the difference was not statistically significant (*P* > 0.05). The ultrafiltration volume after dialysis was 2850 ± 400 mL in the intervention group and 2350 ± 350 mL in the control group. The intervention group was larger than the control group (*P* < 0.05). The details were shown in Table 7.

### 3.6. Comparison on Serous Effusion

The proportion of patients with pleural effusion in the intervention group was 35% before the intervention and 10% after the intervention, and the difference was statistically obvious (*P* < 0.05). The proportion of patients with pleural effusion in the control group was 30% before the intervention and 20% after the intervention, with statistically observable difference (*P* < 0.05). The reduction in pleural effusion patients in the intervention group was significantly greater than in the control group. The details were shown in Table 8.

### 3.7. Comparison of Nursing Satisfaction

The satisfaction questionnaires of the two groups of patients after each dialysis were collected. After integration, it was found that the number of satisfactions in the intervention group was 625, and the satisfaction rate was 97.66%; while the number of satisfactions in the control group was 420, and the satisfaction rate was 65.63%. The satisfaction of the intervention group was obviously higher with statistical difference (*P* < 0.05). The details were shown in Table 9.

## 4. Discussion

ESRD refers to the end stage of various chronic kidney diseases, which is previously called the late stage of uremia. In recent years, the diagnostic criteria for the disease are also changing due to the continuous changes in disease guidelines. Currently, chronic kidney disease stage 5 is end-stage renal disease [18]. Dialysis is often used clinically to reduce the burden on the kidneys, so as to relieve the patient's condition. Dialysis can be clinically divided into two types: hemodialysis and peritoneal dialysis. Both dialysis modes have advantages and disadvantages, but comprehensive hemodialysis has fewer disadvantages. Prehemodialysis often leads to complications such as dialysis imbalance syndrome. Patients will experience nausea, vomiting, dizziness, headache, and even intolerance to hemodialysis. Other patients may have allergic reactions to the dialyzer or dialysis water, and hypotension in hypertensive patients may occur. For patients with late hemodialysis, dialysis-related amyloidosis may occur [19, 20]. Long-term dialysis patients are prone to gastrointestinal bleeding, cerebral hemorrhage, etc. due to the use of anticoagulants, and some patients may have heart failure due to circulatory instability caused by hemodialysis. For peritoneal dialysis patients, peritoneal dialysis-related peritonitis is prone to occur, and the patient presents with abdominal pain, chills, fever, etc., and severe patients may lead to septic shock [21]. Peritoneal dialysis patients are prone to abdominal distension due to the instillation of peritoneal dialysis fluid in their stomachs, and chest tightness may occur after the diaphragm is on the stage [22]. Hemodialysis in the hypotension state is easy to aggravate the patient's hypotension state after the dialysis starts to draw blood [23]. Symptoms of hypoperfusion of systemic organs may occur, such as cardiac ischemia such as palpitations and chest tightness, cerebral ischemia such as dizziness and headache, peripheral circulation ischemia symptoms of numbness of the limbs, and severe hypotension shock [24]. In these cases, the doctor may return the blood to the patient in advance. In this way, the dialysis is insufficient, the patient's toxin and water excretion are significantly reduced, and there will be accumulation of toxins and capacity in the body. In addition, the blood drawn from some patients in the hypotension state is also prone to coagulation in the pipeline, which also affects the dialysis adequacy of the patient and the effect of dialysis [25]. Among them, the occurrence of hypotension in dialysis is considered to be caused by the reduction of effective circulating blood volume due to the ultrafiltration rate and ultrafiltration volume being greater than and bearing the range. In addition, studies have found that high dialysate temperature, low sodium dialysate, acetate dialysate, etc. can promote the occurrence of hypotension during dialysis. Elevated parathyroid hormone levels, bioincompatibility and allergic reactions, and decreased vasopressin can also promote inappropriate vasodilation, resulting in hypotension during dialysis [26].

CRRT is to replace the renal function of patients with acute renal failure by circulating blood through a continuous bradycardia hemofilter and to improve the morbidity through the following effects [27]. It can relieve pulmonary edema and edema, secure the infusion space by removing water from the blood (water removal), and improve the symptoms of pulmonary edema and edema. At the same time, by removing water, the space (infusion space) for dripping the drug into the blood can be guaranteed. Maintaining electrolyte balance can maintain blood pH and electrolyte balance quickly and for a long time. In addition, it should remove the metabolic wastes such as urea and Cre and disease-related substances and eliminate the low-molecular-weight metabolic wastes such as urea and Cre accumulated in the blood. In addition, it can also remove medium molecular weight substances in the range of 20,000 to 30,000 molecular weights such as inflammatory mediators. These substances contain disease-related humoral factors, and the clearance of these substances contributes to the improvement of morbidity [28]. Its treatment modes include the following four. First, continuous veno-venous hemofiltration (CVVH): the filtration pump applies negative pressure from the outside of the hollow fiber and uses the principle of filtration to remove the water and metabolic waste in the blood as filtrate. Second, continuous veno-venous hemodialysis (CVVHD): the dialysate flows from the outside of the hollow fiber, and the metabolic waste is removed by the principle of dispersion. Third, continuous veno-venous hemodiafiltration (CVVHDF) requires fluid replacement and dialysate and uses two principles of filtration and dispersion to remove water and metabolic waste. The pipeline combination is more complicated, but the solute removal performance can be adjusted by adjusting the filtration flow rate and the dialysate flow rate, so that the solute removal performance is between the two modes of CVVH and CVVHD. Four, slow continuous ultrafiltration (SCUF), which uses the same filtration principle as the CVVH mode, discharges water and metabolic waste as filtrate, and is suitable for the treatment of pulmonary edema and edema caused by congestive heart failure and accompanied by lack of urine. Clinically, CRRT intervention can be considered for patients with indications for renal replacement therapy and any of the following conditions: severe acute kidney injury, hemodynamic instability, risk of transport, inability to tolerate other renal replacement therapy (such as intermittent hemodialysis or peritoneal dialysis, and continuous removal of water from the body is required [29]. CRRT has no absolute contraindications, relative contraindications include inability to establish vascular access, severe low, or solute renal or nonrenal disease. Metabolic waste is removed with the movement of water, and electrolytes are removed at the same time, so to maintain electrolyte balance, it is necessary to add fluids. In addition, from small molecular weight substances to medium molecular weight substances in the molecular weight range of 20,000 to 30,000, it can be effectively removed [30].

Existing studies suggest that reducing the incidence of hypotension in patients with dialysis hypotension can be achieved by controlling dry body weight, reducing the intake of watery foods in the daily diet, and limiting the intake of salt, soy sauce, and various preserved foods; changing the dialysis mode; actively treating complications; and rationally applying antihypertensive drugs [31]. In the introduction of individualized nursing, it is pointed out that moderate exercise and psychological guidance can also be added. Therefore, this work integrated the above practices in the content design of individualized nursing strategies and applied them to the nursing of the research subjects. It was compared with the routine nursing, and the nursing effects were analyzed. The results showed that the probability of hypotension during dialysis in the intervention group was lower than that in the control group, and the probability of early termination of dialysis due to hypotension was also lower than that in the control group. The reason is that compared with routine care, individualized care is more detailed in monitoring the patient's condition and incorporates relevant measures to prevent hypotension in patients, so the probability of hypotension is significantly reduced. In the intervention group, the cases of early termination due to discomfort caused by hypotension were significantly reduced, which indirectly improved the effectiveness of the treatment. BUN and Cre are important clinical indicators reflecting renal function. The higher the level, the more serious the renal failure. The results of the work showed that the levels of BUN and Cre in the two groups were decreased to a certain extent compared with those before the intervention, and the decrease of blood urea nitrogen and creatinine in the intervention group was significantly greater than that in the control group. It indicates that the renal function recovery of patients is better under individualized care. Dry body weight, also known as target body weight or ideal body weight, refers to the body weight when the patient has neither water or sodium retention nor dehydration, that is, the body weight when the water metabolism is balanced, that is, the desired body weight at the end of dialysis [32]. In this work, the proportion of water growth during dialysis in the intervention group was greater than that in the control group, the patients with good water control in the intervention group were significantly more than those in the control group, and the amount of ultrafiltration after dialysis in the intervention group was also greater than that in the control group. It means that individualized nursing based on a health science-based diet and strict fluid control can help patients achieve ideal body weight. Long-term dialysis patients are prone to serous effusion due to hypoalbuminemia, infection, and water retention. The satisfaction of the intervention group was significantly higher than that of the control group, indicating that the overall treatment of the patients from the disease itself, daily diet, exercise, and psychology will increase the patients' enthusiasm for treatment and enhance the treatment effect.

## 5. Conclusion

This work compared the effect of individualized nursing and routine nursing in the treatment of ESRD with refractory hypotension using CRRT. The results showed that individualized nursing can reduce the occurrence of dialysis hypotension, help patients achieve ideal body weight, and reduce the occurrence of serous cavity effusion. In addition, the overall satisfaction of patients was high, which can help improve the clinical treatment effect. However, due to the limited sample size of the work, the next step was to expand the research scope and increase the research volume to ensure the accuracy of the research results.

## Figures and Tables

**Figure 1:** Technical route.

**Figure 2:** Flowchart of CRRT.

**Table 1:** Specific contents of individualized nursing.

Measures	Specific contents
Condition nursing	Nursing staff should pay close attention to the changes in the patient's condition. For dialysis patients, it was necessary to regularly observe the changes of vital signs, ask more about the patient's feeling, and detect abnormal changes in the patient's condition in time. It should monitor vital signs once per hour for general patients, and once every 15-30 minutes for critically ill patients to detect the aura symptoms and typical symptoms of hypotension in time, such as yawning, palpitation, nausea, vomiting, and cold sweats. In addition, it should timely inform the dialysis doctor of various changes in the dialysis process and give corresponding treatment.
Dietary guidance	Dialysis patients should strengthen nutrition, improve anemia, and eat high-quality high-protein, low-sodium, and vitamin-rich foods to prevent hypoproteinemia. It should inform the patients and their families to strictly limit the intake of sodium salt and water during dialysis, increase body weight by no more than 3%-5% of body weight, and avoid rapid ultrafiltration, and ultrafiltration of water per hour does not exceed 1% of the body weight. It was not advisable to eat during dialysis. If the condition requires, it should inform the patient that eating during hemodialysis was best within 1-2 hours of the start of dialysis. At this time, the solute and water removed by dialysis only account for 20%-40% of the expected target, which had little effect on peripheral effective circulating blood volume and would not cause blood pressure to drop.
Exercise program	Firstly, postural adaptation exercise should be taken: it should keep the patient in a concave lying position, raise the upper body by 30°, place a soft pillow under the feet, raise it by 15°, and train twice a day, and each training time is 20-30 minutes. Secondly, it should turn over regularly: an alarm clock was placed on the bedside of the hemodialysis treatment, and the alarm clock would ring once every 2 hours. After hearing the alarm, the patient used the healthy limb to grasp the bed rail and perform the ipsilateral turning movement. Nursing staff need to monitor during exercise to ensure that the turning movement does not affect the patency of the pipeline and monitor it effectively. Thirdly, according to the actual situation of the patient, acupuncture was mainly based on aerobic exercise, such as walking and playing Taijiquan. The specific exercise time and amount depended on the patient's tolerance. In addition, it should avoid large movements during exercise.
Psychological nursing	Compared with other treatments, hemodialysis is more likely to cause anxiety, fear, and other adverse emotions in patients, which not only increases the psychological burden but also is not conducive to the treatment of the disease, increasing the probability of hypotension. It can provide targeted psychological care according to the actual situation of the patient, explain the knowledge of the disease to the patient, eliminate the patient's fear of the disease, assist the patient to vent their negative emotions, and maintain a good psychological state. Nursing staff increased the number and time of visits, communicated with patients as much as possible, encouraged, and comforted patients more, and kept patients in the best condition.

**Table 2:** Comparison on basic data of patients.

Item	Intervention group	Control group	*t*/*χ*^2^	*P*
Age	57.13 ± 3.78	56.98 ± 2.67	0.056	0.735
Gender			0.018	0.987
Males	11	12		
Females	9	8		
Course of disease	9.31 ± 2.96	9.28 ± 4.13	0.127	0.396
Number of weekly dialysis	2.79 ± 0.56	2.81 ± 0.13	0.421	0.213

**Table 3:** Comparison on incidence of hypotension and early termination of dialysis.

Group	Times pf hypotension	Incidence of hypotension	Times of early termination of dialysis	Incidence of early termination of dialysis
Intervention group	60	9.38%	0	0
Control group	220	34.38%	120	18.75%
*χ* ^2^	59.673		27.164	
*P*	0.000		0.000	

**Table 4:** Comparison of renal function in intervention group before and after intervention.

Indicators	Intervention group		*t*	*P*
	Before intervention	After intervention		
BUN (mmol/L)	28.46 ± 7.31	15.14 ± 7.56	4.128	0.048
Cre (umoL/L)	360.67 ± 141.84	149.12 ± 140.32	4.063	0.030

**Table 5:** Comparison of renal function before and after intervention in the control group.

Indicator	Control group		*t*	*P*
	Before intervention	After intervention		
BUN (mmol/L)	27.72 ± 7.65	18.32 ± 6.23	4.241	0.007
Cre (umoL/L)	361.68 ± 132.86	169.52 ± 110.67	5.013	0.041

**Table 6:** Comparison of results of weight gain as a percentage of body weight.

Time	Intervention group		Control group		*χ* ^2^	*P*
	<10%	>10%	<10%	>10%		
Before intervention	600 (93.75%)	40 (6.25%)	587 (91.72%)	53 (8.28%)	2.376	0.312
After intervention	630 (98.44%)	10 (1.56%)	598 (93.45%)	42 (6.56%)	27.869	0.000

**Table 7:** Comparison on targeted ultrafiltration volume before dialysis and ultrafiltration volume after dialysis.

Ultrafiltration volume	Intervention group	Control group	*t*	*P*
Targeted ultrafiltration volume before dialysis	3100 ± 500	3000 ± 400	1.545	0.128
Ultrafiltration volume after dialysis	2850 ± 400	2350 ± 350	18.517	0.000

**Table 8:** Comparison on serous effusion before and after the intervention.

Pleural effusion	Intervention group (20 cases)	Control group (20 cases)
Before intervention	7 (35%)	6 (30%)
After intervention	2 (10%)	4 (20%)
*χ* ^2^	10.564	9.708
*P*	0.006	0.007

**Table 9:** Comparison on nursing satisfaction.

Group	Satisfied	General	Unsatisfied	Satisfaction
Intervention group	568	57	15	97.66%^∗^
Control group	212	208	220	65.63%

Note: compared with the control group, the difference was statistically notable (*P* < 0.05).

## Data Availability

The datasets used and analyzed during the current study are available from the corresponding author upon reasonable request.
